# Effects of UCP4 on the Proliferation and Apoptosis of Chondrocytes: Its Possible Involvement and Regulation in Osteoarthritis

**DOI:** 10.1371/journal.pone.0150684

**Published:** 2016-03-02

**Authors:** Zhongming Huang, Junhua Li, Shaohua Du, Guangnan Chen, Yiying Qi, Ligang Huang, Luwei Xiao, Peijian Tong

**Affiliations:** 1 Department of Orthopaedic Surgery, Xiaoshan Chinese Medical Hospital, Hangzhou, China; 2 Department of Orthopaedic Surgery, Affiliated Jiangnan Hospital of Zhejiang Chinese Medical University, Hangzhou, China; 3 Zhejiang Chinese Medical University, Hangzhou, China; 4 Institute of Orthopaedics and Traumatology of Zhejiang Province, Hangzhou, China; 5 Department of Orthopedic Surgery, the Second Affiliated Hospital, School of Medicine, Zhejiang University, Hangzhou, China; 6 Department of Orthopaedic Surgery, the First Affiliated Hospital of Zhejiang Chinese Medical University, Hangzhou, China; University of Maryland School of Medicine, UNITED STATES

## Abstract

Reactive oxygen species (ROS)-induced chondrocytes apoptosis plays a key role in osteoarthritis (OA) pathogenesis. Uncoupling protein 4 (UCP4) can protect cells against oxidative stress via reducing ROS production and cell apoptosis. Here, silencing of UCP4 in primary chondrocytes significantly inhibited cell survival, but induced ROS production and cell apoptosis. UCP4 mRNA of cartilage tissues was decreased in osteoarthritis patients, which was negatively correlated with synovial fluid (SF) leptin concentration. Moreover, leptin treatment (5, 10 and 20 ng/ml) of primary cultured chondrocytes significantly decreased mRNA and protein levels of UCP4, but increased ROS production and cell apoptosis in a dose-dependent manner. The effects of leptin treatment (20 ng/ml) on chondrocytes was partially reversed by ectopic expression of UCP4. More importantly, intraarticularly injection of UCP4 adenovirus remarkably alleviate OA progression and cell apoptosis in a rat OA model induced by anterior cruciate ligament transection (ACLT). In conclusion, UCP4, whose expression was suppressed by leptin, may be involved in the ROS production and apoptosis of chondrocytes, thus contributing to the OA pathogenesis.

## Introduction

Osteoarthritis (OA), one of the most common forms of degenerative joint disease, leads to pain and disability. Approximately 250 million people have OA of the knee (3.6% of the population) in the world [1]. OA is mainly characterized by the degeneration and loss of joint cartilage, which results in the development of bony spurs and cysts at the margins of the joint [2]. The mature articular cartilage matrix has no blood or nerve supply, and the only cells in cartilage, chondrocytes, show little metabolic activity, thus natural cartilage repair is limited. Recent studies have demonstrated the key role of chondrocytes in the degeneration/loss of cartilage and suggested that chondrocytes are target cells for OA therapy.

During the development of OA, chondrocytes exhibit increased apoptosis, cytokine production and matrix degeneration [3–7]. Reactive oxygen species (ROS) production has been found to increase in OA and ROS is considered as an inducer of chondrocyte apoptosis [8]. Uncoupling protein 4 (UCP4) is predominantly expressed in the brain and belongs to UCPs, which are involved in the protection against oxidative stress via reducing ROS production. UCP4 can protect neurons against oxidative stress and calcium overload by reducing ROS production and cellular reliance on mitochondrial respiration [9]. Pre-treatment with leonurine could protect brain tissue against ischemic injury by increasing UCP4 expression [10]. In preadipocytes, overexpression of UCP4 can promote proliferation and inhibit apoptosis [11]. However, whether UCP4 plays a role in the proliferation, ROS production and apoptosis of chondrocytes and whether UCP4 is also involved in the pathogenesis of OA still remain unclear.

Leptin is a small (16 kDa) adipokine mainly produced by adipocyte, and plays a key role in the regulation of food intake and energy expenditure [12–14]. Chondrocytes can express leptin [15] and overexpression of leptin has been reported in OA patients, which suggests that leptin might be involved in the pathogenesis of OA [15–17]. Previous studies demonstrated that leptin can induce apoptosis of rat adipose tissue [18], human bone marrow stromal cells and gastric cancer cells [19, 20]. Expression of other UCPs, including UCP2 and UCP3 [21–23] was regulated by leptin. However, whether leptin induced the apoptosis of chondrocytes and whether UCP4 is involved in the leptin-induced chondrocyte apoptosis is unknown.

In the present study, we hypothesized that UCP4 played a role in the ROS production, apoptosis and survival of chondrocytes, and its expression was regulated by leptin, which might contribute to the OA pathogenesis. So, we detected ROS, cell apoptosis and survival of rat primary chondrocytes treated with UCP4-specific small interfering RNA (siRNA), as well as measured UCP4 mRNA level of human cartilage and leptin concentration in synovial fluid (SF) of OA patients and healthy donors, in an attempt to uncover the role of UCP4 in the apoptosis of chondrocytes and the pathogenesis of OA.

## Materials and Methods

### Human subjects

The study was approval by the Institutional Review Board of Xiaoshan Chinese Medical Hospital (Hangzhou, China). All subjects gave written, informed consent before participation. We collected synovial fluid (SF) samples and cartilage specimens from 50 individuals (ages 51–72 years) with OA that were at diagnosis and undergoing total knee replacement surgery, respectively. Diagnosis was made by arthroscopy, radiography, assessment of joint fluid and clinical examination. Normal synovial fluid samples and cartilage specimens from 20 healthy donors (ages 33–57 years) without history of joint disease.

### Detection of Leptin concentration in SF

SF samples were centrifuged at 3000 g for 30 min to remove cells and particulate matter. Supernatant was separated and stored at −80°C until analysis for no longer than three weeks. Leptin concentration was measured using leptin radioimmunoassay kit according to manufacturer’s instructions (Millipore, Bredford, MA, USA). Samples were measured in duplicate.

### Small interfering RNAs (siRNAs) and adenovirus production

One siRNA (GGCCCUGUUGGAUUAUAAU, UCP4 siRNA) targeting rat UCP4 mRNA (XM_006244611.2) and a nonsense siRNA were synthesized by GenePharma (Shanghai, China).

The UCP4 expression adenovirus (Ad5-UCP4) was constructed using the Ad-Easy Adenoviral Vector System according to the manufacturer’s instructions (Agilent Technologies, Santa Clara, CA, USA). Adenoviruses were purified by ultracentrifugation in cesium chloride gradient and then quantified.

### Quantitative RT-PCR

Total RNA was extracted from tissue samples using TRIzol reagent (Invitrogen, Carlsbad, CA, USA), and cDNA was synthesized from 2 μg RNA using RevertAid First Strand cDNA Synthesis Kit (Fermentas, Hanover, MD, USA) as per the manufacturer’s instructions. Quantitative RT-PCR was performed on a 7300 Sequence Detector System (Applied Biosystems, Foster City, CA, USA) using the Maxima SYBR Green Master Mix (Thermo, Rockford, IL, USA). Expression level of GAPDH was used as a control. Primers were list in Table 1.

**Table 1:** Primers sequences for quantitative RT-PCR.

Primer	Primer sequence	Size (bp)
UCP4 (Homo sapiens) (NM_001204051.1)	F: 5’-CTACATTGCCCAGTAACC-3’; R: 5’-GATAACGCACTCCTTCTC-3’	232
GADPH (Homo sapiens) (NM_008084.2)	F: 5’-ATCACTGCCACCCAGAAG-3’; R: 5’-TCCACGACGGACACATTG-3’	191
UCP4 (Rattus norvegicus) (NM_001170.1)	F:5’-AGGCGTCTGCTAAAGAAGG-3’; R:5’-CTCTGGCAACTCATCTAAGG-3’	112
GADPH (Rattus norvegicus) (NM_001256799.1)	F: 5’-GTCGGTGTGAACGGATTTG-3’; R: 5’-TCCCATTCTCAGCCTTGAC-3’	181

### Western blot

Protein lysates were prepared from cultured chondrocytes, separated by SDS-PAGE and transferred onto PVDF membranes. After blocking with 5% nonfat milk, the membranes were incubated with primary antibodies overnight at 4°C. Then, the membranes were incubated with a horseradish peroxidase-conjugated secondary antibody (Beyotime, Shanghai, China) at room temperature for 1 h. The blots were visualized using Clarity Western ECL kit (BioRad, Richmond, CA, USA) and scanned. The source of primary antibodies were as follows: anti-UCP4, anti-Bcl-2, anti-Bax and anti-PCNA were purchased from Santa Cruz Biotechnology (Santa Cruz, CA, USA), while anti-cleaved Caspase-3 and anti-GAPDH were from Cell Signaling Technology (Danvers, MA, USA).

### Primary cultures of rat chondrocytes

Rat cartilage was collected from knee joints, immediately dissected and digested with 0.4% type II collagenase solution (Sigma, St. Louis, MO, USA) at 37°C for 5 h. After centrifugation at 1000rpm for 5min, isolated chondrocytes were checked for viability using trypan blue staining. Chondrocytes were then cultured with Dulbecco’s Modified Eagles Medium/Ham’s F-12 medium containing 10% fetal bovine serum and 100 U/ml penicillin–streptomycin (Invitrogen).

### Cell viability assay

The proliferation of chondrocyte cultured in 96-well plates was assessed by the use of the Cell Count Kit-8 (CCK-8, Beyotime). At the indicated time point, CCK-8 solution was added to all wells and incubated for 1 h. The absorbance value of each well at 450 nm was measured.

### Measurement of intracellular ROS level and mitochondrial membrane potential (MMP)

The levels of intracellular ROS and MMP were measured using ROS assay kit (Vigorous Biotech, Beijing, China) and MMP kit (Immunochemistry Technologies, Bloomington, MN, USA) following the manufacture’s protocol, respectively. Briefly, chondrocytes were harvest and stained with 50 μmol/L dihydroethidium (DHE) or 100nM tetra methyl rhodamine methyl 1 ester (TMRM) at room temperature in the dark for 30 min. Then, cells were analyzed on a flow cytometry (BD Biosciences, San Jose, CA, USA).

### Flow cytometric analysis of apoptosis

A flow cytometry apoptosis detection kit (Annexin V- fluorescein isothiocyanate [FITC] / Propidium iodide [PI] kit, BD Biosciences) was used to identify cell apoptosis. Cells were suspended in 100 μl of Annexin V binding buffer and then stained with 10 μl FITC-labeled Annexin V (to detect phosphatidylserine expression on cells undergoing early apoptotosis) and PI (to exclude dead cells) in the dark. After stained for 20 min, the cells were analysis on a flow cytometry (BD Biosciences).

### Treatment of chondrocytes

For UCP4 silencing, chondrocytes were transfected with UCP4 siRNA or nonsense siRNA by using Lipofectamine 2000 (Invitrogen) according to the manufacture’s instruction. After two days, UCP4 mRNA and protein expression was determined by quantitative RT-PCR and Western blotting, respectively. Chondrocyte proliferation was assessed by CCK-8 assay at 0 h, 24 h, 48 h and 72 h after siRNA transfection. Chondrocyte apoptosis was evaluated by at 48 h after siRNA transfection.

For leptin treatment, after reaching confluence, cells were cultured in serum deprived medium for 24 h and were subsequently stimulated with leptin (0–20 ng/ml, Sigma, St. Louis, MO, USA) for two days. Chondrocyte proliferation and apoptosis was assessed by CCK-8 assay and flow cytometric analysis, respectively.

For UCP4 overexpression experiments, chondrocytes cultured in serum deprived medium for 24 h were infected with Ad5 or Ad5-UCP4 at the present of 20 ng/ml leptin. mRNA and protein levels of UCP4, and chondrocyte apoptosis was determined at 48 h after treatment. Cell survival was evaluated at 48 h and 72 h after treatment.

### Rat OA model induced by anterior cruciate ligament transection

The experimental protocol was approved by the Animal Care and Use Committee of Xiaoshan Chinese Medical Hospital. Eighteen adult male SPF Sprague Dawley rats (three months old, weighing approximately 300 g) obtained from Shanghai Lab Animal Research Center (Shanghai, China) were used in the present study. All rats were maintained under a 12-h light/ dark cycle at 25°C with free access to a standard diet and water.

The rats were randomly divided into three groups: Group1, sham-operation (sham); Group 2, OA model injected with control adenovirus (Ad5); Group 3, OA model injected with Ad5-UCP4. In Group 2 and Group 3, after rats were anesthetized with 10% chloral hydrate in phosphate-buffered saline (PBS), the knee joints were shaved and disinfected with povidone iodine. Anterior cruciate ligament transection (ACLT) was performed via an incision on the medial aspect of the right knee joint capsule as described previously [24]. Complete transection of the ligament was confirmed by a positive anterior drawer test. In Group 1 (sham-operated group), the wounds were closed after the opening of the joint space and subluxation of the patella.

After surgery on day 0, 7 and 14, rats in Group 2 and Group 3 were intraarticularly injected in the ACLT knees with 3 × 10^7^ pfu control adenovirus (Ad5) and UCP4 adenovirus (Ad5-UCP4), respectively. Rats in Group 1 were given no treatment. Ten weeks after surgery, rats were sacrificed under anesthesia. After the knees were disarticulated, the joints were cut. A portion of samples were snap-frozen, and other samples were fixed in 10% neutral buffered formalin, decalcified in 10% formic acid for 7 days, and paraffin-embedded. Five-μm-thick articular cartilage sections were then cut, deparaffinized and stained with Safranin-O/fast green. The state of the articular cartilage tissue was evaluated by the OARSI scoring method [25]. TUNEL was performed to determine cell apoptosis according to the manufacturer’s instructions (Roche, Germany).

### Statistical analysis

All experiments were performed in triplicate and data are expressed as the mean ± SD. All calculations were performed using the Graphpad Prism software (version 6.0, San Diego, CA, USA). Data were analyzed by student’s t test. Correlation coefficients were calculated by Pearson rank correlation (r). A two-sided P value less than 0.05 was considered as statistically significant.

## Results

### Silencing of UCP4 induces ROS production and apoptosis of rat chondrocytes

Previous studies reported that UCP4 can protect brain tissues from injury via reducing ROS [9, 10], and overexpression of UCP4 can promote proliferation and inhibit apoptosis of preadipocyte [11]. In order to explore the functions of UCP4 on chondrocytes, we decreased its expression by transfection with specific siRNA. Obvious decreases in mRNA and protein levels of UCP4 were observed in rat chondrocytes treated with UCP4-specific siRNA (Fig 1A–1C, P <0.001), while nonsense siRNA transfection has no effect on UCP4 expression when compared with non-treated cells (Mock). Cell proliferation at 48 h and 72 h after UCP4 siRNA transfection was significantly decreased (Fig 1D, P <0.05), which was accompanied by an increase of ROS (Fig 1E, P <0.001) and the early apoptosis rate of chondrocytes (Fig 1F, P <0.001). These data suggested the survival-promoting and apoptosis-inhibitory functions of UCP4 on chondrocytes.

**Fig 1:** UCP4-specific siRNA induced apoptosis of rat chondrocytes. (A-C) Rat chondrocytes were treated with UCP4-specific siRNA for 48 h. mRNA and the protein level of UCP4 were detected using real-time PCR (A) and western blotting assay (B, C). UCP4 expression in control chondrocytes without treatment (Mock) was fixed at 1.0. (D) Cell proliferation was detected in siRNA treated and untreated chondrocytes by CCK-8 assay. Results of cell growth were normalized to the initial cell numbers (100%). (E, F) Chondrocytes were transfected with indicated siRNA for 48 h. Intracellular ROS and cell apoptosis rate was analyzed on a flow cytometry. *P <0.05 and ***P <0.001 versus Nonsense siRNA-treated cells.

### UCP4 mRNA expression was decreased in human OA cartilage

To determine whether the expression of UCP4 mRNA was decreased in OA patients, we collected cartilage tissues from 50 OA patients and 20 healthy donors and performed quantitative RT-PCR analysis. As shown in Fig 2A, UCP4 mRNA was lower in OA cartilage tissues than in normal tissues (P<0.0001). We then re-analyzed expression data of 33 OA and 7 healthy cartilage from NCBI Gene Expression Omnibus database (GEO, GSE57218) [26], and confirmed the downregulation of UCP4 mRNA in OA cartilage (Fig 2B, P<0.0001). The mRNA levels of UCP1, UCP2, UCP3S (UCP3 short form) and UCP3L (UCP3 long form) showed no significant differences between OA and healthy cartilage tissues (S1 Fig). These findings suggested a unique role of UCP4 in OA.

**Fig 2:** UCP4 mRNA was negatively correlated with leptin concentration. (A) UCP4 mRNA expression in cartilage tissues of osteoarthritis patients (n = 50) and health donors (n = 20) was evaluated by quantitative RT-PCR. (B) UCP4 expression analysis based on GSE57218 dataset. (C) Leptin concentrations in SF were measured by using radioimmunoassay kit. (D) Pearson correlation analysis between UCP4 mRNA and leptin SF concentration (P<0.0001).

### UCP4 mRNA level in human cartilage was negatively correlated with leptin concentration in human SF

Leptin was reported increased in the SF of OA patients and may involve in the pathogenesis of OA [15–17]. We then detected the SF concentration of leptin by using a radioimmunoassay kit. The SF concentration of leptin was significantly increased in OA patients when compared with the healthy donors (Fig 2C, P<0.0001). Further correlation analysis showed that UCP4 mRNA level in human cartilage was negatively correlated with the leptin concentration in SF (Fig 2D, P<0.0001).

### Leptin inhibited UCP4 gene expression and cell proliferation, and induced cell apoptosis

To determine whether leptin was involved in the suppression of UCP4 expression in OA cartilage, we treated rat chondrocytes with recombinant leptin and found that leptin decreased mRNA and protein levels of UCP4 in a concentration-dependent manner (Fig 3A–3C, P <0.05). These data suggested that UCP4 may be controlled by leptin at the transcriptional level.

**Fig 3:** Leptin modulated UCP4 expression, cell proliferation and cell apoptosis. (A, B, C) Rat chondrocytes were treated with recombinant leptin (0–20 ng/ml) for 48 h. Then, the mRNA and protein level of UCP4 of chondrocyte cultures was detected. (D) Rat chondrocytes were treated with recombinant leptin (0–20 ng/ml) and cell proliferation was detected. Results of cell growth were normalized to the initial cell numbers (100%). (E, F) Rat chondrocytes were treated with recombinant leptin (0–20 ng/ml) for 48 h, and ROS and cell apoptosis was analyzed. *P <0.05, **P<0.01 and ***P <0.001 versus non-treated cells (0). #P <0.05, ##P<0.01 and ###P <0.001 versus 5 ng/ml leptin-treated cells. +P <0.05 and ++ P<0.01versus 10 ng/ml leptin-treated cells.

Moreover, leptin treatment suppressed cell proliferation (Fig 3D), but induced ROS production (Fig 3E) and cell apoptosis (Fig 3F) in a concentration-dependent manner. The most obvious effects were observed at the dosage of 20 ng/ml, which was chosen for the following assays.

To further investigate whether leptin exerted functions on chondrocytes trough UCP4, UCP4 was overexpressed in chondrocytes via adenovirus transduction in the present of leptin. As displayed in Fig 4A–4C, leptin treatment significantly decreased UCP4 expression both in mRNA and protein levels, while UCP4 adenovirus (Ad5-UCP4) transduction remarkably increased UCP4 expression. The apoptosis promoting and survival inhibitory effects of leptin on chondrocytes were obviously attenuated by ectopic expression of UCP4 (Fig 4D–4F). To investigate whether cell apoptosis was associated with mitochondrial dysfunction, we analyzed mitochondrial membrane potential (MMP) changes in chondrocytes. As shown in Fig 4G, leptin treatment significantly reduced the MMP, which was partially rescued by UCP4 overexpression. These data suggested that UCP4 expression affected cell apoptosis through the intrinsic pathway.

**Fig 4:** Ectopic expression of UCP4 reversed the effects of leptin on the proliferation and apoptosis of chondrocytes. Rat chondrocytes were infected with control adenovirus (Ad5) or UCP4 adenovirus (Ad5-UCP4) in the present of 20 ng/ml leptin. (A, B, C) At 48 h after treatment, the mRNA and protein level of UCP4 of chondrocyte cultures was detected. (D) At 48h and 72h of treatment, cell survival was analysis with CCK-8 assay. (E, F, G) At 48 h after treatment, ROS, cell apoptosis and MMP was analyzed. **P<0.01 and ***P <0.001 versus non-treated cells (Mock). #P <0.05, ##P<0.01 and ###P <0.001 versus 20 ng/ml leptin and Ad5-treated cells.

### Ad5-UCP4 transduction remarkably attenuated OA in a rat model

To further explore the functions of UCP4 on OA in vivo, we established a rat OA model by ACLT [27]. Rats were intraarticularly injected in the ACLT knees with either control adenovirus (Ad5) or UCP4 adenovirus once per week for three consecutive weeks. Ten weeks after surgery, cartilage tissues were collected for histological examination by using Safranin-O/fast green staining. Histological examination results showed that serious degenerative features of OA cartilage, including loss of surface lamina and depletion of chondrocytes, were observed in OA group, which proved the successful establishment of OA model (Fig 5A). In contrast, Ad5-UCP4-treated rats showed significantly attenuated cartilage degeneration. Results of TUNEL assay showed that cells undergoing apoptosis was significantly increased in OA group, while treatment with Ad5-UCP4 notably reduced ALCT surgery-induced cell apoptosis. Consistent with the above results, UCP4 expression was lower in OA model group than in sham-operation group. Ad5-UCP4 treatment significantly increased UCP4 expression (Fig 5B–5D). These data suggested the therapeutic effects of UCP4 on OA.

**Fig 5:** Treatment with UCP4 adenovirus attenuated OA progress in a rat model. (A) Evaluation of histological changes and cell apoptosis in the cartilages by Safranin-O/fast green and TUNEL staining, respectively. OARSI score from three groups of rats (n = 6) was shown. Scale bar: 100 μm. (B, C, D) The mRNA and protein level of UCP4 in rat cartilage tissues were detected. (E) Expression of Cleaved-Caspase-3, Bax, Bcl-2 and PCNA was evaluated by Western blot. **P<0.01 and ***P <0.001 versus sham-operated group (Sham). #P <0.05, ##P<0.01 and ###P <0.001 versus ACLT surgery and Ad5-treated group (OA+Ad5).

We also detected the protein expression of apoptosis-related genes and PCNA in the cartilage tissues. ACLT surgery led to a notable increase in the expression of apoptosis promoting protein (Bax and cleaved-Caspse-3), and a notable decrease in the expression of anti-apoptosis protein (Bcl-2) and proliferation-related protein (PCNA). Ad5-UCP4 treatment significantly attenuated the effects of ACLT surgery on the expression of above proteins (Fig 5E). These data indicated that UCP4 may exert therapeutic effects through inhibiting the apoptosis and promoting the proliferation of chondrocytes.

## Discussion

It is well-known that ROS-induced chondrocytes apoptosis plays a key role in OA pathogenesis. UCPs belongs to a family of nuclear-encoded mitochondrial carriers [28], which are able to decrease ROS production and alter mitochondrial functions [29]. Leptin, a critical factor during OA pathogenesis [15–17], has been reported to regulate the expression of some UCPs, including UCP2 and UCP3 [21–23]. However, there is no study investigated the association between leptin and UCP4 until now. In the present study, we found that UCP4 was associated with ROS production, apoptosis and survival of chondrocytes, and its expression was inhibited by leptin. UCP4 expression was decreased in OA patients, which was negatively related with leptin concentration in SF. Additionally, ectopic expression of UCP4 significantly suppressed disease progression of experimental OA.

Firstly, suppressing UCP4 expression resulted in an obvious decrease in cell survival, and a notable increase in apoptosis of primary cultured chondrocytes (Fig 1), which was consistent with the previous study in preadiopocytes [11]. These findings suggest that UCP4 plays a critical role in the apoptosis and survival of chondrocytes. As chondrocyte is the only cellular component in cartilage, we speculate that UCP4 might further be an essential player in maintaining cartilage function.

Leptin was suggested to play a role in OA pathogenesis [15–17]. Previous studies have investigated the effect of leptin on UCPs expression. Recombinant leptin treatment was found to up-regulate UCP2 mRNA in pancreatic islets [23], increased UCP2 expression in epididymal fat tissue of old rats, whereas it decreased UCP2 expression in that of young rats [22]. Intravenous or intracerebroventricular infusion of leptin was associated with a decrease in UCP2 mRNA in white adipocyte tissue (WAT) and UCP3 mRNA in skeletal muscle [21]. Re-analysis of NCBI GEO database (GSE57218) [26] indicated that there was no significant difference in the mRNA levels of UCP1, UCP2, UCP3S and UCP3L between OA and healthy cartilage tissues (S1 Fig), whereas UCP4 mRNA was significantly lower in OA cartilage tissues than in healthy cartilage tissues (Fig 2B). Phylogenic analysis showed that mammalian UCP1, UCP2 and UCP3 seem to form one subgroup, whereas UCP4 belongs to a different group [28]. Our findings suggested a unique role of UCP4 in OA pathogenesis. Therefore, we then focused our study on UCP4. Here, we found a negative correlation between UCP4 mRNA and leptin levels in human samples (Fig 2). *In vitro* experiment further demonstrated that mRNA and protein expression of UCP4 in primary cultured chondrocyte was suppressed by leptin treatment (Fig 3). Our study firstly demonstrated the regulated role of leptin on UCP4 expression. Moreover, increasing evidence implied that leptin can induce cell apoptosis [19, 20]. Here, our data showed that leptin can induce apoptosis of primary cultured chondrocytes through down-regulating UCP4 expression (Figs 4 and 5), although further investigation on the mechanism how leptin affect UCP4 expression is required.

Furthermore, our *in vivo* OA model experiments showed that intraarticularly injection of UCP4 adenovirus significantly attenuated OA and cell apoptosis, which suggested the therapy value of UCP4 in OA (Fig 5).

In conclusion, UCP4 played a critical role in the ROS production and apoptosis of chondrocytes. UCP4 expression was suppressed in OA patients, and negatively correlated with leptin level. Meanwhile, leptin could suppressed mRNA and protein levels of UCP4. Accordingly, we speculate that leptin might be involved in the suppression of UCP4 gene expression in OA, which would probably contribute to OA pathogenesis.

## Supporting Information

S1 Fig UCP1, UCP2, UCP3S (UCP3 short form) and UCP3L (UCP3 long form) expression analysis based on GSE57218 dataset. (DOCX)
